The article "Circ‐TCF4.85 silencing inhibits cancer progression through microRNA‐486‐5p‐targeted inhibition of ABCF2 in hepatocellular carcinoma" was retracted in 2023. Reasons: duplicated images; signs of a paper mill; unreliable results or conclusions.

# Circ‐TCF4.85 silencing inhibits cancer progression through microRNA‐486‐5p‐targeted inhibition of *ABCF2* in hepatocellular carcinoma

**DOI:** 10.1002/1878-0261.12603

**Published:** 2020-01-10

**Authors:** Jun Gao, Chao Dai, Xin Yu, Xiang‐Bao Yin, Fan Zhou

**Affiliations:** ^1^ Department of Hepatobiliary and Pancreatic Surgery The Second Affiliated Hospital of Nanchang University China

**Keywords:** ATP‐binding cassette subfamily F member 2, circ‐TCF4.85, hepatocellular carcinoma, invasion, microRNA‐486‐5p, migration

## Abstract

The current study aimed to explore the role of the circular RNA circ‐TCF4.85 and its downstream target microRNA‐486‐5p (miR‐486‐5p) in hepatocellular carcinoma (HCC) development. Circ‐TCF4.85 was detected to be highly expressed in HCC tissues. Next, we found that silencing of circ‐TCF4.85 repressed HCC cell proliferation, invasion, and migration, while enhancing apoptosis. In addition, biotin‐coupled probe pull‐down and miRNA capture assays, as well as fluorescence *in situ* hybridization, confirmed that circ‐TCF4.85 could bind to miR‐486‐5p. In rescue experiments, miR‐486‐5p had the potential to eliminate the tumor‐suppressive effects of circ‐TCF4.85 knockdown in HCC. Moreover, miR‐486‐5p was shown to target *ABCF2* gene, which was positively regulated by circ‐TCF4.85. Finally, nude mice subcutaneously injected with si‐circ‐TCF4.85‐transfected HCC cells presented with inhibited xenograft tumor formation *in vivo*. Taken together, our results reveal that silencing of circ‐TCF4.85 suppresses HCC progression via miR‐486‐5p‐targeted inhibition of *ABCF2*.

## Graphical abstract

A potential mechanism of circ‐TCF4.85 was implicated in the occurrence of hepatocellular carcinoma (HCC) via regulation of *ABCF2*. In HCC cells, circ‐TCF4.85 bound to microRNA‐486‐5p (miR‐486‐5p) that targeted and negatively regulated *ABCF2*. Overexpression of circ‐TCF4.85 reduced the expression of miR‐486‐5p, and then increased that of *ABCF2*, thus promoting proliferation, migration, and invasion while suppressing the apoptosis of HCC cells.

**Abbreviations**
ABC: ATP‐binding cassette
ABCF2: ATP‐binding cassette subfamily F member 2
AFP: α‐fetoprotein
ANOVA: analysis of variance
circRNA: circular RNA
DAPI: 4',6‐diamidino‐2‐phenylindole
DMEM: Dulbecco’s modified Eagle’s medium
FISH: fluorescence *in situ* hybridization
GAPDH: glyceraldehyde‐3‐phosphate dehydrogenase
HBV: hepatitis B virus
HCC: hepatocellular carcinoma
IHC: immunohistochemistry
L: length
miRNA or miR: microRNA
MUT: mutant
ncRNA: noncoding RNA
PIK3R1: phosphoinositide‐3‐kinase, regulatory subunit 1 (alpha)
ROC: receiver operating characteristic
RT‐qPCR: reverse transcription‐quantitative polymerase chain reaction
TBST: Tris‐buffered saline Tween‐20
TCGA: The Cancer Genome Atlas
V: volume
W: width
WT: wild‐type

## 1 Introduction

Hepatocellular carcinoma (HCC) is the 5th most frequently occurring cancer and the most ubiquitous liver malignancy throughout the world, with rising incidence and mortality rates (Mittal and El‐Serag, 2013; Tao *et al.*, 2011). With more than 700 000 people being diagnosed with HCC every year, HCC represents a major health concern around the world (Bruix *et al.*, 2014). Unfortunately, the prognosis of HCC is unfavorable and even presents with high recurrence rates as a result of high frequency of intrahepatic and extrahepatic metastases (Yuan *et al.*, 2014). Adding to the plight of the condition, only a third of patients are eligible to receive curative treatments (Han *et al.*, 2017). Therefore, it is trivial to discover and test potential targets for the prognosis and treatment of HCC. In recent years, several noncoding RNA (ncRNA), such as long ncRNA and microRNA (miRNA or miR), have been identified as potential targets for HCC therapies (Li *et al.*, 2017; Xiong *et al.*, 2010). However, the specific involvement of circular RNA (circRNA) in HCC remains unclear.

Circular RNA represent a family of naturally occurring ncRNA that are widespread in the human eukaryotic transcriptome (Memczak *et al.*, 2013). The circRNA exert critical roles in regulating gene expressions by acting as sponges of miRNA, which helps to facilitate the increasing repertoire of the regulatory functions in gene expression (Hansen *et al.*, 2013; Li *et al.*, 2015). The biological effects of circRNA have attracted much attention over the last few decades, especially for the initiation and development of cancers (He *et al.*, 2018). The initial microarray analysis in the current study indicated that there were unregulated levels of circ‐TCF4.85 in HCC. Moreover, Huang *et al.* have revealed that circRNA‐100338 serves as a potential biomarker in the diagnosis and prognosis of HCC via regulation of miR‐141‐3p (Huang *et al.*, 2017). MicroRNA also represents a type of ncRNA capable of repressing mRNA translation or reducing mRNA stability by binding to the 3′UTR of their target mRNA (Ma *et al.*, 2015; Otsuki *et al.*, 2015). In addition, miRNA serve as paramount regulators in a variety of biological processes such as cellular proliferation, migration, apoptosis, and even tumorigenesis (Xiao *et al.*, 2015). Interestingly, previous evidence has documented downregulated levels of microRNA‐486‐5p (miR‐486‐5p) in HCC and further indicated that miR‐486‐5p inhibits the progression of HCC via negative regulation of its target gene, phosphoinositide‐3‐kinase, regulatory subunit 1 (alpha) (*PIK3R1*) (Huang *et al.*, 2015). Moreover, analyses from the website http://www.microRNA.org revealed that ATP‐binding cassette subfamily F member 2 (*ABCF2*) is a target gene of miR‐486‐5p. ATP‐binding cassette (ABC) transporter superfamily, known as the largest transporter gene family, has been implicated in the transportation of specific molecules across lipid membranes in living organisms (Liu *et al.*, 2011). Furthermore, high levels of the ABC subfamily G member 2b are also found in liver (Ren *et al.*, 2015). Based on the above‐mentioned literature, we employed human normal liver cell lines and HCC cell lines as well as xenograft in nude mice to explore the possible effects of circ‐TCF4.85 on HCC cellular processes via mediating miR‐486‐5p and *ABCF2*.

## 2 Materials and methods

### 2.1 Ethics statement

The current study was carried out with the approval of the Ethics Committee of the Second Affiliated Hospital of Nanchang University (No. 201312004). Signed informed consent was obtained from all participants prior to tissue collection, which was in accordance with the Declaration of Helsinki. Further, animal experiments were performed in line with the protocols approved by the Institutional Animal Research Committee of the Second Affiliated Hospital of Nanchang University (China).

### 2.2 Microarray‐based circRNA expression profiling

Gene expression datasets of HCC‐related circRNA were downloaded from the Gene Expression Omnibus (GEO) database (https://www.ncbi.nlm.nih.gov/geo/). The Affy package of r language was applied for standard pretreatment for datasets (Gautier *et al.*, 2004). Next, Limma package of r language was adopted to verify the differentially expressed circRNA. After correction, the *P*‐value was expressed as *adj.P.Val*. |log2FC|> 1.5 and circRNA with *adj.P.Val* < 0.05 was regarded as differentially expressed circRNA. A map of the obtained circRNA was then plotted. We further speculated on the potential regulation mechanism of circ‐TCF4.85 using the CircNet database available at http://circnet.mbc.nctu.edu.tw/. In addition, the Cancer Genome Atlas (TCGA) database available at http://ualcan.path.uab.edu/index.html was used for analysis of gene expression regulated by circRNA as well as the survival curve (Chandrashekar *et al.*, 2017) .

### 2.3 Study subjects

Hepatocellular carcinoma and adjacent normal tissues were harvested from 46 patients who were diagnosed with HCC (31 males and 15 females; aged 32–76 years) who underwent surgical treatment at the Second Affiliated Hospital of Nanchang University between 2013 and 2016. None of the patients received any drug treatment prior to sample collection. All tissue samples were subsequently immersed in liquid nitrogen and stored at −80° C for later use. The follow‐up duration was 3 years.

### 2.4 Cell culture

The human 293T cell, human normal liver cell L‐02, human HCC cell lines SMMC‐7721, Huh‐7, and SK‐Hep‐1, and hepatoblastoma‐derived cell line HepG2 were incubated in Dulbecco’s modified Eagle’s medium (DMEM; Thermo Fisher Scientific, Inc., Waltham, MA, USA) containing 10% FBS (Thermo Fisher Scientific, Inc.), 100 mg·mL^−1^ streptomycin, and 100 U·mL^−1^ penicillin. All cells were cultured in a 37° C incubator with 5% CO_2_ in air and saturated humidity.

### 2.5 RNA isolation and quantitation

The total RNA content of the cells was extracted using a TRIzol kit (Shanghai Haling Biotechnology Co., Ltd., Shanghai, China). The extracted RNA underwent reverse transcription to synthesize complementary DNA following the instructions of a reverse transcription kit (TransGen Biotechnology, Co., Ltd., Beijing, China). Next, reverse transcription‐quantitative polymerase chain reaction (RT‐qPCR) was performed according to the instructions of the SYBR® Premix Ex TaqTM II Kit (Takara Biotechnology Co., Ltd., Dalian, China) using the ABI PRISM® 7500 System (ABI Company, Oyster Bay, NY, USA). The primers were synthetized by the Beijing Genomics Institute (China) (Table 1). The calculation in relation to the ratio of the gene expression between two groups was conducted using the $2^{-\Delta \Delta C_{t}}$ method, and the employed formula was as follows: △△C*_t_* = △C*_t_*_experimental group_ − △C*_t_*_control group_. C*_t_* value represented the amplification cycles when the value reached the set threshold (Zhang *et al.*, 2016a). The expression of miR‐486‐5p was determined using the TaqMan miRNA Assay according to the manufacturer’s instructions (Thermo Fisher Scientific, Inc.) with U6 serving as internal reference.

**Table 1:** Primer sequences of related genes for RT‐qPCR. F, forward; R, reverse.

Gene	Sequence (5'‐3')
miR‐486‐5p	F: ACACTCCAGCTGGGTCCTGTACTGAGCTGCCC
	R: CTCAACTGGTGTCGTGGAGTCGGCAATTCAGTTGAGCCCCGAG
U6	F: CTCGCTTCGGCAGCACA
	R: AACGCTTCACGAATTTGCGT
circ‐TCF4.85	F: GTGTACTTGGATGAGTTTCGTCG
	R: TTGCCAC ATTAAAGGCAGCTC
*ABCF2*	F: GAGGTTTCACTGGGAGCAAGATC
	R: CTGTAGCGTCTTCTCCTTGCTC
GAPDH	F: GACTCATGACCACAGTCCATGC
	R: AGAGGCAGGGATGATGTTCTG

### 2.6 Western blot analysis

A Bio‐Rad DC Protein Assay kit (Ewell Biotechnology Co., Ltd., Guangzhou, China) was employed to determine the concentration of proteins. The proteins were then separated with SDS/PAGE and subsequently transferred onto a polyvinylidene fluoride membrane. The membranes were immersed in 1 × Tris‐buffered saline Tween‐20 (TBST) with 5% skimmed milk and gently shaken for 2 h to block nonspecific binding. Subsequently, the membranes were incubated with the following diluted primary antibodies: rabbit anti‐human ABCF2 (dilution ratio of 1 : 2000, ab86178; Abcam Inc., Cambridge, UK) or rat anti‐human glyceraldehyde‐3‐phosphate dehydrogenase (GAPDH; dilution ratio of 1 : 5000, ab8245; Abcam Inc.) at 4° C overnight. After TBST wash, the membranes were incubated for 1 h with the secondary antibody, goat anti‐rabbit IgG (dilution ratio of 1 : 20 000, ab6721; Abcam Inc.). Three rinses with TBST followed.

### 2.7 3‐[4,5‐Dimethylthiazol‐2‐yl]‐2,5‐diphenyl tetrazolium bromide (MTT) assay

Eight days after incubation, the cells were harvested and inoculated in 96‐well plates (at a density of 1 × 10^4^ cells per well). Each well was subjected to incubation with 20 μL MTT solution (Shanghai Fortuneibo‐tech Co., Ltd., Shanghai, China) for 4 h, followed by centrifugation. After removal of supernatant, 100 µL dimethyl sulfoxide was added to each well. The samples were oscillated on a micro‐oscillator for 10 min. After complete dissolution of the purple crystals, the optical density values at 490 nm were measured using a microplate reader.

### 2.8 Clonogenic assay

Cells were planted in 6‐well plates (at a density of 400 cells per well), and cultured in DMEM supplemented with 10% FBS. After 2 weeks, the cells underwent fixation with methanol and staining with 0.1% crystal violet. Finally, the newly formed colonies were imaged and counted.

### 2.9 Scratch test

Cells in each group were planted in 6‐well plates (at a density of 2.5 × 10^4^ cells per cm^2^). After 24‐h culture, the medium was absorbed. Scratches were evenly made using a 10 μL sterile disposable pipette. Thereafter, the samples were rinsed twice with PBS, and further incubated in RPMI 1640 culture medium with 10% FBS. The wound healing was observed at 0 hour and 48 hours after scratching at the same position. Three duplicated wells were set. HCC cell migration was calculated using the following formula: scratch distance = (the number of cells at scratched area at *T*_24_ − the number of cells at scratched area at *T*_0_)/the number of cells at scratched area at *T*_0_ × 100%.

### 2.10 Transwell assay

The apical chamber of a Transwell chamber (aperture of 8 μm; Costar, Cambridge, MA, USA) was covered with the Matrigel (BD Biosciences, San Jose, CA, USA). After drying, the transfected cells (about 1 × 10^4^) were suspended in 200 μL serum‐free culture medium and inoculated in the apical chamber. The medium with 10% FBS was subsequently added to the basolateral chamber. Cells were incubated in a 37° C incubator with 5% CO_2_ for 48 h. Thereafter, the cells in the apical chamber were wiped off using cotton swabs, and those on the surface of basolateral chamber were fixed in methanol and stained with 0.1% crystal violet, followed by photographing and observation under a microscope (×200; Olympus Optical Co., Ltd., Tokyo, Japan).

### 2.11 Flow cytometry

A total of 1 × 10^6^ cells at the logarithmic phase of growth were harvested, rinsed twice with PBS and fixed with 70% cold EtOH. The cells were then stained with 1 mL propidium iodide (50 μg·mL^−1^; Becton, Dickinson and Company, Franklin Lakes, NJ, USA) in dark conditions for 30 min. A FACSCalibur flow cytometer (Becton, Dickinson and Company) was employed to detect cell cycle, which was then analyzed using modfit software (BD Biosciences San Jose, CA, USA).

Next, 1 × 10^6^ cells at the logarithmic growth phase were harvested and rinsed twice with cold PBS. After being suspended with 1× Annexin buffer, the cells were incubated with 5 μL Annexin‐V‐FITC (Becton, Dickinson and Company, Rutherford, NJ, USA) at room temperature for 10 min devoid of light. Thereafter, a flow cytometer was utilized to detect the apoptosis of HCC cells.

### 2.12 Biotin‐coupled probe pull‐down assay

Biotin‐coupled probe of circ‐TCF4.85 with miR‐486‐5p binding region was designed. The probe sequence was TCTCATGGCCCAGTGTAAAA. A total of 1 × 10^7^ cells were rinsed in precooled PBS, followed by immersion in the lysis buffer and incubation with a 3 μg biotinylated probe for 2 h. The cell lysate was incubated with streptavidin‐loaded magnetic beads [Life Technologies Corporation (Gaithersburg, MD, USA); Thermo Fisher Scientific (Waltham, MA, USA)] for 4 h to pull down the biotin‐coupled RNA complex. The magnetic beads subsequently underwent five washes with lysis buffer, and the binding miRNA was isolated from complex using a TRIzol agent and analyzed by RT‐qPCR.

### 2.13 Biotin‐coupled miRNA capture

The 50 μm biotinylated miRNA mimic (GenePharma, Shanghai, China, sequence GCCCTTCATGCTGCCCAG) was transfected into approximately 2 × 10^6^ cells at 50% confluence. After transfection for 24 h, the cells were harvested, rinsed with PBS, and lysed in the lysis buffer. After washing, 50 μL of streptavidin‐coated magnetic beads were sealed for 2 h and added into each reaction tube in an attempt to pull down the biotin‐coupled RNA complex. The beads were then rinsed five times with lysis buffer. TRIzol LS (Life Technologies Corporation, Thermo Fisher Scientific, Inc.) was used to recycle the RNA interacting with the specificity of miRNA. The circ‐TCF4.85 enrichment was analyzed and evaluated using RT‐qPCR and agarose gel electrophoresis, respectively.

### 2.14 Fluorescence *in situ* hybridization (FISH)

The circ‐TCF4.85 sequence and miR‐486‐5p specific probes were subjected to FISH. The cy5‐labeled probe showed specificity to circ‐TCF4.85, whereas the farm‐labeled probe showed specificity to miRNA. The nuclei were stained with 4',6‐diamidino‐2‐phenylindole (DAPI). All procedures were conducted according to the instructions of FISH kit (GenePharma). All images were obtained under a Zeiss LSM880 NLO confocal microscope (Leica Microsystems, Mannheim, Germany).

### 2.15 Dual‐luciferase reporter gene assay

The binding region between ABCF2 and miR‐486‐5p was predicted using the biological prediction website http://www.microRNA.org. Firstly, we constructed ABCF2 3′UTR gene fragments that were inserted into the pMIR‐reporter (Promega, Madison, WI, USA), after which complementary sequences with mutant (MUT) binding sites were designed based on the wild‐type (WT) ABCF2 seed sequences. Next, the sites were constructed in the pMIR‐reporter plasmid. The luciferase reporter plasmids ABCF2‐WT and ABCF2‐MUT that were correctly sequenced were cotransfected with miR‐486‐5p mimic and mimic negative control (NC) into HEK‐293T cells (Beinuo Life Science Co., Ltd., Shanghai, China), respectively. After transfection for 48 h, the cells were harvested and lysed. The luciferase activity was detected using the Dual‐Luciferase Reporter Assay System (Promega).

### 2.16 Tumorigenicity assay in nude mice

The Huh‐7 cells were transfected with circ‐TCF4.85 or empty vectors. About 1 × 10^7^ transfected cells were subcutaneously injected into the armpit of 30 female BALB/c athymic nude mice (aged 5–6 weeks, weighing 16–20 g), with 15 nude mice in each group. The width (W) and length (L) of tumors were measured using calipers every week to record tumor growth, and the tumor volume (V) was calculated using the following equation: V = (W^2^ × L)/2. At the 4th week after injection, the nude mice were euthanized and tumors were excised and weighed.

### 2.17 Immunohistochemistry (IHC)

Paraffin‐embedded samples were sliced into 4‐μm‐thick sections. The sections were dewaxed, dehydrated, and incubated in a 3% H_2_O_2_ incubator (Sigma‐Aldrich, Chemical Co., St. Louis, MO, USA) at 37° C for 30 min. After PBS rinsing, the sections were boiled in 0.01 m citric acid buffer at 95° C for 20 min, cooled down to the room temperature, and rinsed with PBS. Subsequently, the sections were blocked with normal goat serum working fluid at 37° C for 10 min. The sections were incubated with rabbit anti‐mouse ABCF2 (dilution ratio of 1 : 100, ab87318; Abcam Inc.), followed by incubation with the biotin‐labeled goat anti‐rabbit secondary antibody. Three different fields (×200) in each section photographed by the Japan Nikon Image analysis were selected to calculate the number of positive cells. The criterion of the IHC results was as follows: ABCF2 (the percentage of positive cells more than 25%) with obvious brown and brown‐yellow particles in the cytoplasm. The positive rate was calculated with the number of positive cells divided by total cells (Feng *et al.*, 2015).

### 2.18 Statistical analysis

Statistical analyses were conducted using the spss 21.0 software (IBM Corp., Armonk, NY, USA). Measurement data were depicted as mean ± SD. Comparisons between two groups were analyzed by independent‐samples *t*‐test with Welch’s correction. Data normality was tested by Shapiro–Wilk test. Data conforming to normal distribution among multiple groups were analyzed by one‐way analysis of variance (ANOVA). Least significant difference test was employed for pairwise comparison among groups. Comparisons of skewed data were conducted using nonparametric Kruskal–Wallis test. Comparisons of data at different time points were analyzed by repeated‐measures ANOVA. A value of *P* < 0.05 was indicative of statistical significance.

## 3 Results

### 3.1 Circ‐TCF4.85 and *ABCF2* are upregulated in HCC

Initially, we employed the r software to screen the differentially expressed circRNA, which revealed that circ‐TCF4.85 was upregulated in the http://www.ncbi.nlm.nih.gov/geo/query/acc.cgi?acc=GSE94508 dataset (Fig. 1A). In addition, we adopted the CircNet website (http://circnet.mbc.nctu.edu.tw/) to further speculate on the possible regulation mechanisms of circ‐TCF4.85 (Fig. 1B) and then applied the TCGA database to analyze the potential regulatory genes, which demonstrated that *ABCF2* was highly expressed in HCC and shared a correlation with HCC prognosis (Fig. 1C,D).

**Figure 1:** Highly expressed circ‐TCF4.85 and *ABCF2* in HCC and circ‐TCF4.85 exhibits a potential diagnostic significance in HCC. (A) A heat map of the top 10 differentially expressed circRNA in the http://www.ncbi.nlm.nih.gov/geo/query/acc.cgi?acc=GSE94508 dataset, in which the abscissa refers to the sample number and the ordinate refers to differentially expressed circRNA; the upper right histogram refers to color gradation and each rectangle represents the expression level of one sample. (B) The potential regulation mechanisms of circ‐TCF4.85 in HCC. (C) The expression patterns of *ABCF2* in HCC. (D) Survival curve of *ABCF2* in HCC. (E) Circ‐TCF4.85 expression patterns in HCC tissues and adjacent normal tissues detected using RT‐qPCR. (F) circ‐TCF4.85 expression patterns in the L‐02, SMMC‐7721, Huh‐7, SK‐Hep‐1, and HepG2 cell lines detected by RT‐qPCR. (G) ROC curve of circ‐TCF4.85 expression differentiating HCC patients from normal controls. * *P* < 0.05, compared with adjacent normal tissues or L‐02 cells. Data are expressed as mean ± SD. Comparisons between the adjacent normal tissues and HCC tissues were analyzed using paired *t*‐test in (E) (*n* = 46) and those among multiple groups were analyzed by one‐way ANOVA. The experiment was repeated three times.

We recorded the clinicopathological characteristics of 46 patients including gender, age, hepatitis B virus (HBV) infection, tumor size, vascular invasion, distant metastasis, and clinical staging. The results are shown in Table 2. The mean plasma α‐fetoprotein (AFP) level in those patients was 807.49 ± 64.22 µg·L^−1^. RT‐qPCR was applied to detect the expression patterns of circ‐TCF4.85 in 46 adjacent normal and HCC tissues, the results of which demonstrated that HCC tissues exhibited elevated levels of circ‐TCF4.85 (Fig. 1E). In addition, circ‐TCF4.85 was expressed at higher levels in the four HCC cell lines (SK‐Hep‐1, Huh‐7, HepG2, and SMMC‐7721) compared with the normal cancer cell line L‐02 (Fig. 1F). The upregulated expression of circ‐TCF4.85 in both HCC cells and tissues was consistent with the aforementioned microarray‐based circRNA expression analysis. Next, we plotted a receiver operating characteristic (ROC) curve for the differentiating value of circ‐TCF4.85 in HCC patients from normal controls as depicted in Fig. 1F. The area under the curve was calculated to be 0.891 (95% confidence interval = 0.820–0.962; *P* < 0.001). With an optimal threshold of 1.8425, circ‐TCF4.85 exhibited a sensitivity of 86.8% and a specificity of 87.0%, suggesting a good predictive value of circ‐TCF4.85 expression in the diagnosis of HCC.

**Table 2:** Clinicopathological characteristics of patients with HCC.

Characteristics	Pooled population (*n* = 46)
Gender	
Female	31
Male	15
Age (years)	
< 65	41
≥ 65	5
HBV infection	
Positive	34
Negative	12
Tumor size (cm)	
> 5	20
3–5	26
Vascular invasion	
Yes	17
No	29
Distant metastasis	
Yes	15
No	31
Clinical staging	
I–II	35
III	11

### 3.2 Depleted circ‐TCF4.85 impedes the viability, migration, and invasion of HCC cells *in vitro*

RT‐qPCR was adopted to detect the expression patterns of circ‐TCF4.85 and linear TCF4.85 to verify that circ‐TCF4.85 was a circRNA. The results revealed decreased circ‐TCF4.85 expressions in si‐circ‐TCF4.85‐transfected cells, whereas no significant differences were detected in relation to linear TCF4.85 expression (Fig. 2A). It was suggested that in the current study, the regulatory effect was exerted by circ‐TCF4.85 rather than linear TCF4.85. Due to elevated levels of circ‐TCF4.85 in HCC cell lines and tissues, we aimed to investigate the potential role of circ‐TCF4.85 by downregulating its expression in Huh7 cells. MTT assay, clonogenic assay, scratch test, and Transwell assay were carried out in a bid to detect the viability, colony formation, migration, and invasion capacities of HCC cells, respectively. HCC cell viability (Fig. 2B), colony number (Fig. 2C,D), migration (Fig. 2E,F), and invasion (Fig. 2G,H) were found to be suppressed in the absence of circ‐TCF4.85. The results revealed that circ‐TCF4.85 knockdown hindered the cell proliferation, invasion and migration capacities *in vitro* in HCC.

**Figure 2:** Downregulation of circ‐TCF4.85 represses the viability, migration, and invasion of HCC cells *in vitro*. (A) Circ‐TCF4.85 and linear TCF4.85 expression patterns in si‐circ‐TCF4.85‐transfected cells determined using RT‐qPCR. (B) HCC cell viability in the absence of circ‐TCF4.85 assessed using MTT assay. (C) Colony formation of HCC cells transfected with si‐circ‐TCF4.85 using clonogenic assay. (D) Colony‐forming cell number in response to si‐circ‐TCF4.85 transfection. (E) HCC cell migration in response to si‐circ‐TCF4.85 transfection measured using scratch test. (F) Wound width in response to si‐circ‐TCF4.85 transfection. (G) HCC cell invasion in response to si‐circ‐TCF4.85 transfection evaluated using Transwell assay. (H) The quantitative analysis of invasive cell number. * *P* < 0.05, compared with the NC group. Data were expressed as mean ± SD; comparisons between two groups were analyzed using unpaired *t*‐test, and those among multiple groups were analyzed by repeated‐measures ANOVA. The experiment was repeated three times.

### 3.3 Depleted circ‐TCF4.85 impedes cell cycle progression and promotes apoptosis of HCC cells

Flow cytometry was employed to detect cell cycle and apoptosis of HCC cells with the aim of elucidating the role of circ‐TCF4.85 in HCC cell cycle and apoptosis. The results displayed that there were more G1 phase‐arrested cells in the absence of circ‐TCF4.85 (Fig. 3A,B), suggesting that si‐circ‐TCF4.85 induced cell cycle arrest. In addition, transfection with si‐circ‐TCF4.85 was found to enhance apoptosis of HCC cells (Fig. 3C,D). The data suggested that circ‐TCF4.85 silencing promoted apoptosis in HCC *in vitro*.

**Figure 3:** Circ‐TCF4.85 knockdown impedes cell cycle progression at the G1 phase and enhances apoptosis of HCC cells. (A) Cell cycle progression in response to si‐circ‐TCF4.85 transfection measured by flow cytometry. (B) Proportion of cells at the G1 phase in response to circ‐TCF4.85 knockdown. (C) Apoptosis in HCC cells in response to si‐circ‐TCF4.85 transfection detected by flow cytometry. (D) Apoptotic rate of HCC cells after circ‐TCF4.85 knockdown. *P < 0.05, compared with the NC group; Data were expressed as mean ± SD and analyzed using unpaired *t*‐test. The experiment was repeated three times.

### 3.4 Circ‐TCF4.85 specifically binds to miR‐486‐5p

The microarray analysis (Starbase V2.0, Circinteractome) predicted that circ‐TCF4.85 may bind to miR‐486‐5p in HCC cells. Subsequent RT‐qPCR demonstrated that circ‐TCF4.85 was pulled‐down and enriched using circ‐TCF4.85 specific probes in HCC cells (Fig. 4A). The specific enrichment of circ‐TCF4.85 and miR‐486‐5p was observed in the biotin‐coupled RNA complex that was pulled down using beads (Fig. 4B), which proved that circ‐TCF4.85 can directly bind to miR‐486‐5p. The binding of circ‐TCF4.85 to miR‐486‐5p was further verified using biotin‐coupled miRNA capture and FISH assays. Similarly, more circ‐TCF4.85 was captured in biotin‐coupled miR‐486‐5p, indicating that miR‐486‐5p could bind with circ‐TCF4.85 (Fig. 4C). Moreover, FISH analysis revealed colocalization of circ‐TCF4.85 and miR‐486‐5p in the cytoplasm of HCC (Fig. 4D). Thus, it was corroborated that circ‐TCF4.85 can bind to miR‐486‐5p.

**Figure 4:** Circ‐TCF4.85 binds to miR‐486‐5p. (A) Circ‐TCF4.85 enriched by specific probes detected by RT‐qPCR. (B) miR‐486‐5p enriched by circ‐TCF4.85 specific probe detected by RT‐qPCR. (C) Expression of circ‐TCF4.85 captured by biotin‐coupled miR‐486‐5p detected by RT‐qPCR. (D) Colocalization of circ‐TCF4.85 and miR‐486‐5p revealed by FISH assay (×400). *P < 0.05, compared with the biotin NC group. Data were expressed as mean ± SD, and comparisons between two groups were analyzed using unpaired *t*‐test. The experiment was repeated three times.

### 3.5 MicroRNA‐486‐5p reverses the promoting effects of circ‐TCF4.85 on viability, migration, and invasion of HCC cells

Subsequently, we detected the miR‐486‐5p expression patterns in 46 adjacent normal and HCC tissues and found that miR‐486‐5p was downregulated in HCC tissues (Fig. 5A). The correlation analysis displayed a negative correlation between miR‐486‐5p and circ‐TCF4.85 (Fig. 5B). Next, we evaluated the potential mechanism of miR‐486‐5p in HCC in cells transfected with miR‐486‐5p mimic in the presence of circ‐TCF4.85 by conducting rescue experiments. The results revealed that the viability, invasion, migration, and colony formation capacities of HCC cells overexpressing circ‐TCF4.85 were all significantly increased, whereas they were reversed by miR‐486‐5p mimic‐mediated upregulation of miR‐486‐5p (Fig. 5C–I). Flow cytometry data displayed that HCC cells overexpressing circ‐TCF4.85 presented with an increased number of cells at the G2 phase, whereas miR‐486‐5p mimic suppressed the increase of G2 phase‐arrested HCC cells caused by elevated circ‐TCF4.85 (Fig. 5J,K). In addition, cell apoptosis results by flow cytometry demonstrated that circ‐TCF4.85 overexpression inhibited cell apoptosis, whereas miR‐486‐5p mimic reversed the inhibitory role of circ‐TCF4.85 in cell apoptosis (Fig. 5L,M). The above‐mentioned findings suggested that miR‐486‐5p eliminated the promoting effects of circ‐TCF4.85 on HCC cell colony formation, proliferation, invasion, and migration capacities.

**Figure 5:** MicroRNA‐486‐5p overexpression disrupts the promoted HCC cell viability, colony‐forming ability, migration, and invasion induced by circ‐TCF4.85. HCC cells were transfected with miR‐486‐5p mimic in the presence of circ‐TCF4.85. (A) MicroRNA‐486‐5p expression patterns in HCC tissues and adjacent normal tissues detected by RT‐qPCR. (B) Correlation analysis of circ‐TCF4.85 and miR‐486‐5p. (C) HCC cell viability in each group detected using MTT assay. (D) HCC cell colony formation ability in each group detected using clonogenic assay. (E) Colony‐forming cell number in each group. (F) HCC cell migration in each group detected using scratch test. (G) Migration distance in each group. (H) HCC cell invasion in each group detected using Transwell assay (×400). (I) Invasive cell number in each group. (J) Cell cycle progression detected by flow cytometry. (K) Proportion of cells at G1, S, and G2 phases in each group. (L) Cell apoptosis in each group detected by flow cytometry. (M) Apoptotic rate of HCC cells in each group. *P < 0.05, compared with the NC group; #* P* < 0.05, compared with the circ‐TCF4.85 group. Data were expressed as mean ± SD. Comparisons between adjacent normal tissues and HCC tissues were analyzed using *t*‐test (*n* = 46), and those among multiple groups were analyzed by the one‐way ANOVA or repeated‐measures ANOVA. Correlation analysis between two groups was conducted using Pearson’s correlation analysis. The experiment was repeated three times.

### 3.6 Circ‐TCF4.85 positively regulates *ABCF2*, a target gene of miR‐486‐5p

Next, we performed *in silico* analysis available at microRNA.org in an attempt to detect whether miR‐486‐5p could regulate ABCF2, which revealed the binding sites between miR‐486‐5p and *ABCF2* in HCC (Fig. 6A). Subsequent dual‐luciferase reporter gene assay demonstrated that miR‐486‐5p mimic cotransfection with ABCF2‐wt‐3′‐UTR resulted in a significant decrease in luciferase activity, whereas cotransfection with ABCF2‐mut‐3′‐UTR showed no evident differences (Fig. 6B). In addition, RT‐qPCR was applied to detect the *ABCF2* expression patterns, revealing significantly increased *ABCF2* expression in HCC tissues (Fig. 6C). Furthermore, the correlation analysis manifested that circ‐TCF4.85 presented with a positive correlation with *ABCF2* (Fig. 6D). Additionally, RT‐qPCR was applied to identify the antitumor effect of circ‐TCF4.85 by regulating *ABCF2* via miR‐486‐5p. The findings showed that circ‐TCF4.85 overexpression increased the expression of *ABCF2* (Fig. 6E,F), whereas miR‐486‐5p mimic‐induced elevation of miR‐486‐5p obviously reduced the mRNA and protein levels of *ABCF2* (Fig. 6G,H). The above‐mentioned findings verified that *ABCF2* was directly targeted by miR‐486‐5p. In addition, by conducting circ‐TCF4.85 and miR‐486‐5p gain‐of‐function experiments, we observed that circ‐TCF4.85 partly reversed the inhibitory role of miR‐486‐5p in *ABCF2* (Fig. 6I).

**Figure 6:** Circ‐TCF4.85 positively regulates the expression of *ABCF2*, a target gene of miR‐486‐5p. (A) Bioinformatic analysis of the binding site between miR‐486‐5p and *ABCF2*. (B) The binding of miR‐486‐5p to ABCF2 confirmed by dual‐luciferase reporter gene assay. (C) *ABCF2* mRNA expression patterns in HCC tissues and adjacent normal tissues detected using RT‐qPCR. (D) Correlation analysis of circ‐TCF4.85 and *ABCF2*. (E) *ABCF2* mRNA expression patterns in cells overexpressing circ‐TCF4.85 detected using RT‐qPCR. (F) *ABCF2* protein‐level patterns in cells overexpressing circ‐TCF4.85 using Western blot analysis. (G) *ABCF2* mRNA expression patterns in cells transfected with miR‐486‐5p mimic determined using RT‐qPCR. (H,I) Western blot analysis of ABCF2 protein in cells transfected with miR‐486‐5p mimic or cotransfected with circ‐TCF4.85 and miR‐486‐5p mimic. * *P *< 0.05, compared with the NC group. Data were expressed as mean ± SD. Comparisons between adjacent normal tissues and HCC tissues were analyzed using *t*‐test (*n* = 46), and those among multiple groups were analyzed by the one‐way ANOVA or repeated‐measures ANOVA. Correlation analysis between two groups was conducted using Pearson’s correlation analysis. The experiment was repeated three times.

### 3.7 Depleted circ‐TCF4.85 suppresses xenograft tumor formation *in vivo*

Mice were subcutaneously injected with Huh‐7 cells transfected with si‐circ‐TCF4.85 or its NC to verify the effects of circ‐TCF4.85 on tumor growth *in vivo*. After tumor formation, the tumor volume was measured. Nude mice injected with Huh‐7 cells transfected with si‐circ‐TCF4.85 displayed obviously decreased tumor volume and weight compared with those injected with NC‐transfected Huh‐7 cells (Fig. 7A–C). Western blot analysis further revealed that nude mice injected with Huh‐7 cells transfected with si‐circ‐TCF4.85 exhibited evidently reduced expressions of *ABCF2* at protein level (Fig. 7D,E). Furthermore, IHC results demonstrated that the nude mice injected with si‐circ‐TCF4.85‐transfected Huh‐7 cells showed evidently reduced *ABCF2* expressions (Fig. 7F,G). The obtained findings indicated that silencing of circ‐TCF4.85 reduced the *ABCF2* expression and inhibited xenograft tumor formation in nude mice.

**Figure 7:** Downregulation of circ‐TCF4.85 inhibits xenograft tumor formation in nude mice. (A) Xenograft tumor formation in nude mice. (B) Tumor volume of nude mice. (C) Tumor weight of nude mice. (D,E) Western blot analysis of ABCF2 protein in nude mice injected with NC‐transfected or si‐circ‐TCF4.85‐transfected Huh‐7 cells. (F,G) Representative images of *ABCF2*‐positive cells detected by IHC (×400), and *ABCF2*‐positive rate in nude mice injected with NC‐transfected or si‐circ‐TCF4.85‐transfected Huh‐7 cells. *P < 0.05, compared with the NC group. Data were expressed as mean ± SD. Comparisons between two groups were analyzed using unpaired *t*‐test, and those among multiple groups were analyzed by repeated‐measures ANOVA (*n* = 15). The experiment was repeated three times.

## 4 Discussion

Hepatocellular carcinoma is a major histological subtype among primary liver cancers and the 2nd leading contributor of cancer‐related deaths in China (Chen *et al.*, 2017; Zhang *et al.*, 2016b). Despite sustained efforts by researchers over the last few years, the prognosis of HCC remains poor because of high metastases and recurrence rates (Yuan *et al.*, 2014). The progression of HCC is very intricate, a cascade of epigenetic and genetic alterations regulating the function of proteins post‐translationally, which facilitates metastasis and invasion and leads to worse prognoses (Chen *et al.*, 2011). The current study aimed to explore *the in vivo* and *in vitro* effects of circ‐TCF4.85 regulating miR‐486‐5p and *ABCF2* on HCC initiation and progression. Collectively, our data indicated that depletion of circ‐TCF4.85 upregulated miR‐486‐5p to repress cell proliferation, migration, and invasion capacities, and promote apoptosis via suppression of *ABCF2* in HCC.

Initial results obtained from the current study revealed that circ‐TCF4.85 was extensively expressed in HCC tissues and cell lines and its expression exhibited a diagnostic value. Multiple circRNA have already been documented to be overexpressed in HCC tissues and to participate in the occurrence and progression of HCC (Meng *et al.*, 2017). For instance, hsa_circ_0005075, upregulated in HCC, has been highlighted as a potential HCC biomarker in cancer progression (Shang *et al.*, 2016). Another study uncovered elevated levels of hsa_circ_0016788 in both HCC tissues and cell lines, whereas silencing of hsa_circ_0016788 suppressed tumorigenesis (Guan *et al.*, 2018). In the current study, *in vitro* *and in vivo* experimentation results illustrated that depletion of circ‐TCF4.85 impeded proliferation, invasion, and migration capacities as well as tumorigenicity of HCC cells, but induced cell apoptosis. Similarly, a previous study noted that hsa_circ_0016788 silencing inhibits proliferation and invasion and promotes apoptosis *in vitro*, concomitantly with suppression of tumor growth *in vivo* (Guan *et al.*, 2018). Moreover, Qin *et al.* (2016) stated that circ‐0001649 exerts crucial impacts on tumorigenesis and metastasis of HCC due to its correlation with the occurrence of tumor embolus and tumor size, highlighting circ‐0001649 as a potential target for HCC. Furthermore, silencing of circ‐0067934 has been previously demonstrated to decelerate proliferation, invasion and migration of HCC cells as well as tumor growth, while promoting cell apoptosis (Zhu *et al.*, 2018).

Another key finding obtained from the current study was that circ‐TCF4.85 can bind to miR‐486‐5p. A previous study also confirmed this binding relationship and stated that circ‐001569 competitively binds to miR‐145 and then inhibits its activity (Xie *et al.*, 2016). Circ_0067934 has been found to bind to miR‐545 and consequently suppress its expression (Hu *et al.*, 2019). CircRNA, also known as miRNA sponge, possess the ability to regulate gene expression acting as competing endogenous RNA and also modulate the expression of miRNA‐targeted transcripts in multiple eukaryotes (Xuan *et al.*, 2016). By inhibiting miR‐767‐3p, hsa_circ_0000673 upregulates the *SET* gene, a downstream target of miR‐767‐3p, to stimulate HCC cell proliferation and invasion (Jiang *et al.*, 2018). Another study further revealed that circ_0074027 could bind to miR‐518a‐5p to elevate IL17RD and consequently promote glioblastoma cell growth and invasion (Qian *et al.*, 2019). In the current study, we discovered that miR‐486‐5p could reverse the contributory effects of circ‐TCF4.85 on HCC cell proliferation, invasion, and migration capacities. Accumulating evidence has also implicated aberrantly expressed miRNA in the progression of HCC via their direct control on cell growth and metastasis (Huang *et al.*, 2015). In addition, miR‐486‐5p is poorly expressed in HCC, and functions to inhibit HCC cell growth, invasion, migration, and facilitate apoptosis so as to repress tumor growth via regulation of PIK3R1 and phosphatidylinositol 3‐kinase‐AKT activation (Huang *et al.*, 2015; Zhang *et al.*, 2014). Additionally, miR‐486‐5p acts as a tumor‐suppressive miRNA by negatively regulating oncogenes NEK2 and IGF‐1R (Fu *et al.*, 2017; Youness *et al.*, 2016). *ABCF2* is reported to be correlated with multidrug resistance; it inhibition is responsible for the antitumor role of miR‐122 in HCC (Yahya *et al.*, 2018), suggesting that inhibition of *ABCF2* might suppress cancer development. Our study provides further evidence that circ‐TCF4.85 rescued the miR‐486‐5p‐induced inhibition of its target gene *ABCF2*. Hence, it is reasonable to suggest that silencing of circ‐TCF4.85 inhibits *ABCF2* to retard HCC progression by upregulating miR‐486‐5p.

## 5 Conclusion

In conclusion, the current study provides evidence that circ‐TCF4.85 knockdown upregulates miR‐486‐5p to hinder the cell proliferation, migration, and invasion and induce apoptosis by downregulating the expression of *ABCF2* in HCC, highlighting inhibition of circ‐TCF4.85 as a potential target to prevent the initiation or progression of HCC (Fig. 8). Further studies are warranted in other HCC cell lines to elucidate the specific mechanism of the network in HCC.

**Figure 8:** Potential mechanism of circ‐TCF4.85 implicated in the occurrence of HCC via regulation of *ABCF2*. In HCC cells, circ‐TCF4.85 bound to miR‐486‐5p that targeted and negatively regulated *ABCF2*. Overexpression of circ‐TCF4.85 reduced the expression of miR‐486‐5p, and then increased that of *ABCF2*, thus promoting proliferation, migration, and invasion while suppressing the apoptosis of HCC cells. By contrast, inhibition of circ‐TCF4.85 repressed the elevated the miR‐486‐5p expression, accompanied by decreased *ABCF2* expression, resulting in a decline in the proliferation, migration, and invasion but an increase in the apoptosis of HCC cells.

## Conflict of interest

The authors declare no conflict of interest.

## Author contributions

JG, CD, XY, X‐BY, and FZ designed the study. JG and CD collated the data, conducted data analyses, and produced the initial draft of the manuscript. XY, X‐BY, and FZ contributed to drafting the manuscript. All authors read and approved the final submitted manuscript.
